RETRACTED

# USP22 Protects Against Myocardial Ischemia–Reperfusion Injury via the SIRT1-p53/SLC7A11–Dependent Inhibition of Ferroptosis–Induced Cardiomyocyte Death

**DOI:** 10.3389/fphys.2020.551318

**Published:** 2020-10-21

**Authors:** Shuxian Ma, Linyan Sun, Wenhao Wu, Jiangli Wu, Zhangnan Sun, Jianjun Ren

**Affiliations:** ^1^Department of Anesthesiology, The Second Hospital of Hebei Medical University, Shijiazhuang, China; ^2^Department of Anesthesiology, Qingyun People’s Hospital, Qingyun, China

**Keywords:** ubiquitin specific peptidase 22, myocardial ischemia–reperfusion injury, sirtuin-1, p53, solute carrier family 7 member 11, ferroptosis, cardiomyocyte death

## Abstract

Myocardial ischemia–reperfusion (MI/R) injury is characterized by iron deposition and reactive oxygen species production, which can induce ferroptosis. Ferroptosis has also been proposed to promote cardiomyocyte death. The current study sought to define the mechanism governing cardiomyocyte death in MI/R injury. An animal model of MI/R was established by ligation and perfusion of the left anterior descending coronary artery, and a cellular model of IR was constructed in cardiomyocytes. ChIP assay was then conducted to determine the interaction among USP22, SIRT1, p53, and SLC7A11. Loss- and gain-of-function assays were also conducted to determine the *in vivo* and *in vitro* roles of USP22, SIRT1, and SLC7A11. The infarct size and pathological changes of myocardial tissue were observed using TCC and hematoxylin–eosin staining, and the levels of cardiac function– and myocardial injury–related factors of rats were determined. Cardiomyocyte viability and apoptosis were evaluated *in vitro*, followed by detection of ferroptosis-related indicators (glutathione (GSH), reactive oxygen species, lipid peroxidation, and iron accumulation). USP22, SIRT1, and SLC7A11 expressions were found to be down-regulated, whereas p53 was highly expressed during MI/R injury. USP22, SIRT1, or SLC7A11 overexpression reduced the infarct size and ameliorated pathological conditions, cardiac function, as evidenced by reduced maximum pressure, ejection fraction, maximum pressure rate, and myocardial injury characterized by lower creatine phosphokinase and lactate dehydrogenase levels *in vivo*. Moreover, USP22, SIRT1, or SLC7A11 elevation contributed to enhanced cardiomyocyte viability and attenuated ferroptosis-induced cell death *in vitro*, accompanied by increased GSH levels, as well as decreased reactive oxygen species production, lipid peroxidation, and iron accumulation. Together, these results demonstrate that USP22 overexpression could inhibit ferroptosis-induced cardiomyocyte death to protect against MI/R injury *via* the SIRT1/p53/SLC7A11 association.

RETRACTED

## Introduction

Acute myocardial infarction (AMI) contributes to a large proportion of mortality across the globe. Currently, reperfusion strategies are regarded as the treatment of choice for AMI, but reperfusion is likely to precipitate paradoxical cardiomyocyte dysfunction, namely ischemic reperfusion injury (IRI) (Neri et al., 2017). Myocardial reperfusion is usually implemented either with the application of thrombolytic treatment or primary percutaneous coronary intervention (Yellon and Hausenloy, 2007). These advanced measures possess the ability to swiftly recover blood circulation to the ischemic myocardium to salvage the living myocardium, minimize myocardial infarct size, maintain left ventricular systolic functions, and most importantly, avoid the happen of myocardial failure. However, the recovery of blood flow can bring about additional cardiac damage and complications, in particular, the death of cardiomyocytes, which is regarded as myocardial ischemia–reperfusion (MI/R) injury (Hausenloy and Yellon, 2013).

Additionally, large amounts of iron have been suggested to possibly raise the potential risk of coronary artery diseases (Kobayashi et al., 2018). Recently, a study further illustrated that ferroptosis, which is an emerging concept of iron-dependent cell death, could regulate the fate of chemotherapy, as well as MI/R caused cardiomyopathy (Fang et al., 2019). Ferroptosis accounts for a new category of programmed cell death depicted by iron-dependent aggregation of lipid peroxides to toxic ranges, which distinguishes itself from apoptosis, necroptosis, and autophagy from a morphological, biochemical, and genetic standpoint (Stockwell et al., 2017). Understanding the specific mechanism of ferroptosis-induced cardiomyocyte death could thus prove pivotal to achieve effective attenuation of MI/R injury.

Another focus of the current study, the USP22 protein is a member of the deubiquitinase family, which comprises of more than 70 members (McCann et al., 2020). USP22 has further been correlated with enhanced intestinal tissue regeneration following intestinal I/R injury (Ji et al., 2019). Studies have also shown that USP2a functions as a deubiquitinase, which not only deubiquitinates β-catenin, but also stabilizes it (Kim et al., 2018). Moreover, Lin et al. (2012) reported that USP22 serves as a specific deubiquitinase of NAD-dependent protein deacetylase sirtuin-1 (SIRT1), and this deubiquitination guided stabilization of SIRT1 repressed p53 transcriptional activity and proapoptotic functions. SIRT1, the human ortholog of yeast silence information regulator 2 (SIRT2), is a component of mammalian NAD-dependent sirtuin deacetylases, which carry out roles in catalyzing the process of histone deacetylation together with additional substrates, and confer widespread influence on several processes such as inflammation, aging, mitochondrial biogenesis, cell senescence, apoptosis, and circadian rhythms (Liu et al., 2020). More importantly, depletion of SIRT1 has been reported to exacerbate I/R injury in aged livers (Chun et al., 2018). Furthermore, studies have shown that reduced intestinal expressions of SIRT1 can protect mice against alcohol-induced liver injury by reducing ferroptosis (Zhou et al., 2020). Based on the aforementioned literature, we proposed a hypothesis that USP22/SIRT1 axis may play pivotal roles in ferroptosis-induced cardiomyocyte death, and sought to define its roles in an animal model of MI/R and a cellular model of IR in cardiomyocytes, hoping to highlight a novel targeting approach to MI/R therapy.

RETRACTED

## Materials and Methods

### Ethical Approval

All animal experiment procedures were approved by the Animal Experiment Ethics Committee of The Second Hospital of Hebei Medical University, and extensive efforts were made to minimize the suffering of the included animals.

### Establishment and Grouping of *in vivo* MI/R Animal Model

A total of 84 Sprague-Dawley rats (aged 8 weeks) were adopted for the experiments, which were randomly divided into the three following groups: normal (*n* = 12; rats received no treatment), sham-operated rats (*n* = 12; rats were sham-operated), and MI/R rats (*n* = 60; rats were established as MI/R model). Myocardial MI/R rat models were induced by ligation and perfusion of the left anterior descending coronary artery (LAD). Briefly, the rats were subjected to adaptive feeding for 1 week prior to modeling. The rats were anesthetized by intraperitoneal injection of 1.5% sodium pentobarbital (50 mg/kg) and placed on a temperature-controlled heating pad to expose the LAD, and a 6–0 suture was passed through the LAD to form a slipknot around the LAD. After 30 min of ischemia, the knot was released to restore blood flow. The rats were then sacrificed after 3 or 24 h of reperfusion. At the end of the reperfusion, blood samples were collected, and the myocardial tissues were quickly removed. Meanwhile, the sham-operated rats underwent myocardial exposure after thoracotomy without LAD ligation.

The 60 MI/R rats were classified into the five following groups (12 rats/group): MI/R rats (rats without any other treatment); MI/R rats treated with negative control (NC) rats (rats were injected with the empty adenovirus vector through the right common carotid artery for 7 days, followed by MI/R model construction); MI/R rats treated with overexpressed (oe)-USP22 group (rats were injected with the recombinant adenovirus vector oe-USP22 through the right common carotid artery for 7 days, followed by MI/R model construction); MI/R rats treated with oe-USP22 + short hairpin RNA (sh)-SIRT1 group (rats were injected with the recombinant adenovirus vector oe-USP22 and sh-SIRT1 through the right common carotid artery for 7 days, followed by MI/R model construction); and MI/R rats treated with oe-USP22 + sh-solute carrier family 7 member 11 (SLC7A11) (rats were injected with the recombinant adenovirus vector oe-USP22 and sh-SLC7A11 through the right common carotid artery for 7 days, followed by MI/R model construction). The shRNA (20 μL; 0.8 μg/g) or adenovirus vector was delivered *via* three separate injections (Sun et al., 2017). After 12 h of surgery, six rats in each group were euthanized to isolate the hearts for subsequent experimentation, whereas the cardiac function of the remaining six rats in each group was measured after 2 weeks.

RETRACTED

### Measurement of Infarct Size

After 12 h of I/R injury, rats (*n* = 6/group) were euthanized to determine the area of myocardial necrosis. In brief, the sections were incubated in 2% triphenyltetrazolium chloride (TTC) phosphate buffer (pH 7.4) at 37°C for 30 min, and then fixed with 10% formaldehyde solution for 24 h to enhance color contrast. Subsequently, myocardial tissues were separated for infraction observation. The light red coloration represented ischemic myocardium without infarction, whereas areas with inactive enzymes and infarction remained unstained and appeared pale, whereby grayish-white coloration represented infarcted myocardium. Unstained areas were measured using the ImageJ software to calculate the percentage of grayish-white areas.

### Immunohistochemistry

The myocardial tissue sections were baked at 60°C for 1 h and dewaxed in xylene for 30 min. Subsequently, the sections were dehydrated with gradient alcohol of 95, 80, and 75% for 1 min/each, followed by incubation in 3% H_2_O_2_ (84885, Sigma-Aldrich, San Francisco, CA, United States) at 37°C for 30 min. Thereafter, the myocardial tissue sections were placed in 0.01 M citrate buffer, boiled at 95°C for 20 min, and then allowed to cool down to room temperature. After being sealed in normal goat serum at 37°C for 10 min, the sections were probed with rabbit anti-mouse monoclonal antibody USP22 (ab195289, dilution ratio of 1:100, Abcam, Cambridge, United Kingdom) overnight at 4°C. The sections were then reprobed with rabbit secondary antibody (ab6721, dilution ratio of 1:2,000, Abcam) for 30 min at room temperature. Next, the sections were treated with streptavidin–biotin–peroxidase complex for 30 min and stained with 3 mL of diaminobenzidine (DAB; DA1010; Beijing Solar Science and Technology Co., Ltd.) for 5–10 min. The sections were subsequently counterstained with hematoxylin, sealed, and fixed with neutral resin. Positive cells were represented as brown areas. Three areas of each sample in the experiment were randomly captured using a camera (Leica, Wetzlar, Germany) and analyzed using the ImageJ software.

RETRACTED

### Hematoxylin–Eosin Staining of Myocardial Tissue

Myocardial tissue sections were immersed in hematoxylin for 3–4 min and stained with eosin for 1–2 min. After that, the sections were dehydrated in 80, 90, and 100% ethanol for 3–5 min each, dewaxed with xylene for 3 min, and then sealed with a neutral gel. Five visual fields of view were randomly selected from each stained section, followed by microscopic observation (Olympus, Tokyo, Japan).

### Cell Culture

H9C2 cardiomyocytes were cultured in high-glucose Dulbecco modified eagle medium (DMEM) supplemented with 10% fetal bovine serum (FBS), penicillin (100 U/mL), and streptomycin (100 μg/mL) in a humidified incubator (5% CO_2_, 95% air, 37°C) (Wang et al., 2013). When confluence reached 90%, the cells were passaged. To establish IR models in cardiomyocytes, H9C2 cells were subjected to hypoxia (2 h)/reoxygenation (24 h) (HR). To simulate hypoxia, the culture medium of the cells was renewed with low-glucose DMEM without FBS in a hypoxia incubator (cultured under 5% CO_2_, 95% N_2_, 37°C), followed by conventional reoxygenation. Cells in the control group remained in normal incubators without HR stimulation. Cells were harvested after 24 h to isolate cellular proteins. Ferroptosis was induced by erastin (10 μM) for 8 h before hypoxia (Zhang et al., 2018).

### Hemodynamic Measurement

After 2 weeks of surgery, six rats in each group were adopted to measure cardiac function. Briefly, the rats were anesthetized with 1.5–2% isoflurane. A 1.4-Fr Miller catheter tip micromanometer (SPR-839; Miller Instruments) was inserted into the left ventricle of rats through the right carotid artery. After 15 min of stabilization, the pressure signal and myocardial rate were continuously recorded using an ARIA pressure-volume conductance system with a Powerlab/4SP A/D converter. The cardiac function of rats was then determined by assessment of hemodynamic parameters including reduced maximum pressure, decreased ejection fraction, and decreased maximum pressure rate (dP/dT max).

### Determination of Biochemical Indexes

Serum levels of creatine phosphokinase (CPK) and lactate dehydrogenase (LDH) are regarded as biochemical indices of cardiomyocyte damage. After perfusion, 1 mL of blood was collected from the carotid arteries of the rats and stored at room temperature for 30 min, followed by centrifugation at 2,795 × *g* for 10 min. The upper serum was collected, and the serum levels of CPK (at 450 nm) and LDH (at 340 nm) were measured using a spectrophotometry adhering to the instructions of K777-100 and K726-500 kits, respectively (BioVision Inc., Bioptics, Tucson, AZ, United States). The Olympus AU2700 automatic biochemical analyzer (Beckman Coulter, Tokyo, Japan) was adopted to evaluate the serum levels of LDH and creatinine phosphokinase isoenzyme (CPK-MB).

RETRACTED

### 3-(4,5-Dimethylthiazol-2-yl)-2, 5-Diphenyltetrazolium Bromide Assay

3-(4,5-Dimethylthiazol-2-yl)-2, 5-diphenyltetrazolium bromide (MTT) assay was applied to determine cell viability. In advance, 5 mg/mL MTT was dissolved in phosphate-buffered saline (PBS) and filtered with a sterile filter to ensure sterility. The filtered MTT solution was then wrapped with tin foil in dark conditions and stored in a refrigerator at -20°C to ensure the accuracy of reaction. Cells were collected during the logarithmic phase, and then cell suspension was incubated in a 96-well plate (1 × 10^4^ cells/well) at 37°C in 5% CO_2_. After H9C2 cells were anoxic and reoxygenated, the supernatant was removed and cells were rinsed with PBS and centrifuged again. Next, 180 μL of fresh culture medium was added to each well together with 20 μL of 0.5% MTT solution (5 mg/mL) for incubation for 4 h. After removing the culture medium from each well, 150 μL of dimethyl sulfoxide was added to each well, followed by 10 min shaking to fully dissolve the crystals. The absorbance of each well was measured at a wavelength of 490 nm using a MTT enzyme-linked immunometric meter. Meanwhile, dimethyl sulfoxide wells (medium, MTT) and control wells (cells, drug dissolution medium of the same concentration, culture solution, MTT, dimethyl sulfoxide) were set up, and three sets of wells were set for each group.

### Lipid Peroxidation Assay

H9C2 cells were lysed using a cell lysis buffer (C0481, Sigma, St Louis, MO, United States), and the supernatant was prepared with a thiobarbituric acid (TBA)-glacial acetic acid reagent. After 1 h of incubation at 95°C, the malondialdehyde (MDA)-TBA adduct was colorimetrically quantified using a spectrophotometer at a wavelength of 532 nm. Lipid peroxidation was then determined by measuring the amount of MDA with a lipid peroxidation assay kit (ab118970, Abcam) according to the manufacturer’s instructions.

### Iron Assay

Total iron content in cell lysates was quantified using an iron assay kit (Abcam, ab83366). In short, after reoxygenation, the H9C2 cells were lysed in the iron assay buffer and centrifuged at 16,000 × *g* for 10 min to remove the insoluble matter. Next, 5 μL of iron reducing agent was added to 50 μL of cell samples for total iron (Fe^3+^ and Fe^2+^) analysis. Later, 100 μL of the iron probe solution was added for incubation at 25°C in dark conditions for 60 min. Spectrophotometry was finally adopted to detect the absorbance at a wavelength of 593 nm.

RETRACTED

### Glutathione Detection

To measure total glutathione (GSH) levels and the ratio of the oxidation of GSH to GSH disulfide (GSSG), GSH/GSSG Quantification kits (Donjindo, Kumamoto, Japan) were employed. After reoxygenation, the H9C2 cells were collected and lysed using 10 mM HCl. Next, 5% 5-sulfosalicylic acid (5-SSA) was added to the cells and centrifuged at 8,000 × *g* for 10 min. The 0.5% 5-SSA supernatant was finally collected for detection.

### Reactive Oxygen Species Detection

After reoxygenation, the H9C2 cells were incubated with 2 mL of 10 μM DCFH-DA probe at 37°C in dark conditions for 30 min (Leng et al., 2018). The unbound dye was removed by rinsing with 2% PBS-containing FBS. The sample was then centrifuged at 1,000 rpm for 3 min, and the pellets were resuspended in 500 μL of PBS containing 2% FBS. Measurements were conducted using a FACS Calibur flow cytometer (Becton Dickinson, San Jose, CA, United States). The FlowJo software was finally adopted to measure the fluorescence of each probe. The figure shows the average percentage of positive cells in each total cell ± standard deviation.

### Chromatin Immunoprecipitation (ChIP) Assay

H9C2 cells were cross-linked with 1% formaldehyde for 10 min at room temperature and neutralized by adding glycine to adjust to a final concentration of 0.125 M. After rinsing with PBS twice, the cells were collected and suspended in cold lysis buffer (10 mM Tris-Cl, pH 8.0, 85 mM KCl, 0.5% NP40, 5 mM ethylenediaminetetraacetic acid (EDTA), 0.25% triton, and 1x protease inhibitor). Following incubation on ice for 10 min, the nuclei were collected, resuspended in LB3 buffer and sonicated to obtain 200–50 base pair operator DNA fragments. Magnetic beads coated with p53-specific antibodies or immunoglobulin G (IgG) (control) were then added to the lysate and incubated overnight. The following day, the beads were washed seven times with washing buffer (50 mM HEPES, pH 7.5; 500 mM LiCl; 1 mM EDTA; 1% NP-40; and 0.7% sodium deoxycholate), and once with TE buffer. Protein–DNA complex was finally eluted from the beads.

### Western Blot Analysis

The protein expression patterns of USP22, SIRT1, p53, and SLC7A11 in myocardial tissues and H9C2 cells were examined. The cells were lysed with cell lysis buffer (C0481, Sigma) and incubated at 4°C for 30 min. Following this, the cell lysates were then collected into 1.5 mL EP tubes and centrifuged at 12,000 × *g* at 4°C for 15 min to collect the supernatant. The protein concentration was then determined using a bicinchoninic acid assay protein determination kit (Beyotime Biotechnology, Shanghai, China). After boiling for 5 min, 20 μg of the protein samples was passed through a 10% sodium dodecyl sulfate polyacrylamide gel electrophoresis gel, and then electro-transferred onto a polyvinylidene fluoride membrane (Millipore, Billerica, MA, United States). Subsequently, the membrane was blocked using 5% skimmed milk powder for 1 h, and probed with TBST-diluted rabbit antibody USP22 (ab195289, dilution ratio of 1:1,000, Abcam), mouse antibody SIRT1 (ab110304, dilution ratio of 1:1,000, Abcam), mouse antibody p53 (ab26, dilution ratio of 1:1,000, Abcam), and rabbit antibody SLC7A11 (ab175186, dilution ratio of 1:2,000, Abcam) at 4°C overnight. The membrane was then reprobed with horseradish peroxidase (HRP)-labeled rabbit secondary antibodies (ab6721, dilution ratio of 1:2,000, Abcam) or rat secondary antibodies (ab6728, dilution ratio of 1:2,000, Abcam) at room temperature for 1 h. Enhanced chemiluminescence reagent was adopted for color development (Baoman, Shanghai, China), with rabbit antibody β-actin (ab179467, dilution ratio of 1:4,000) serving as the internal reference. The gray value of each band was analyzed using the ImageJ software, and finally, the ratio of gray levels of the target protein and the internal reference protein band was calculated.

RETRACTED

### Reverse Transcription–Quantitative Polymerase Chain Reaction

Cells were lysed using a Trizol kit (Thermo Fisher, Austin, Texas, United States) to extract the total RNA content from the cells and tissue samples. Ultraviolet-visible spectrophotometry (ND-1000, NanoDrop, United States) was subsequently adopted to detect the quality and concentration of RNA. Total RNA was then extracted using RNeasy Mini kits (Qiagen, Valencia, CA, United States), and mRNA expression was determined by reverse transcription (RT) using a reverse transcription kit (RR047A, Takara, Japan) to obtain complementary DNA (cDNA). Next, the cDNA was used as a template and quantitative polymerase chain reaction (PCR) was performed as per the instructions of SYBR^®^ Premix Ex TaqTM II (Perfect Real Time) kit (DRR081, Takara, Tokyo, Japan). After mixing the sample, RT–quantitative PCR (PCR) was performed with a real-time qPCR instrument (ABI 7500, ABI, Foster City, CA, United States). Glyceraldehyde-3-phosphate dehydrogenase (GAPDH) mRNA levels were used as internal controls to normalize the results. The primers are shown in Table 1. The 2^–ΔΔ*Ct*^ method was adopted and the formula is as follows: ΔΔCT = ΔCt of experimental group—ΔCt of control group, where ΔCt = Ct of target gene – Ct of internal reference gene. Ct indicates the number of amplification cycles that the reaction’s real-time fluorescence intensity needs to pass when it reaches a set detection threshold. At this time, the amplification is increasing at a logarithmic phase.

RETRACTED

**TABLE 1:** Primer sequences used for RT-qPCR.

Genes (Rno)	Primer sequences (5′–3′)
USP22	F:5′-CATGACCCCTTTCATGGCCT-3′
	R:5′-GATGTTCTGGTGACGGGTGT-3′
SIRT1	F:5′-TCATTCTGACTGTGATGACGA-3′
	R:5′-CTGCCACAGTGTCATATCCAA-3′
p53	F:5′-CATGAGCGTTGCTCTGATG-3′
	R:5′-CAGATACTCAGCATACGGATTTCC-3′
SLC7A11	F:5′-GTCCTCTATGTGGAG-AATGA-3′
	R:5′-TCTTGGTCATCATCT-TGGTA-3′
GAPDH	F:5′-AGACAGCCGCATCTTCTTGT-3′
	R:5′-CTTGCCGTGGGTAGAGTCAT-3′

*RT-qPCR, reverse transcription–quantitative polymerase chain reaction; F, forward; R, reverse; USP22, ubiquitin specific peptidase 22; SIRT1, sirtuin-1; SLC7A11, solute carrier family 7 member 11; GAPDH, glyceraldehyde-3-phosphate dehydrogenase.*

### Statistical Analysis

Statistical analyses of the data were performed using SPSS 21.0 (IBM, Armonk, NY, United States) statistical software. Measurement data are presented as mean ± standard deviation from at least three independent experiments. Unless otherwise mentioned, statistical comparisons were performed using unpaired *t* test when only two groups were compared. One-way analysis of variance (ANOVA) followed by Tukey *post hoc* test was adopted when more than two groups were compared. *p* < 0.05 indicated statistical significance.

## Results

### USP22 Protects Against MI/R Injury

To elucidate the molecular mechanism of MI/R injury, we established a rat model of MI/R, and examined myocardial infarction by TTC staining (Supplementary Figure 1A). In addition, rat serum CPK and LDH levels were examined to verify the successful construction of MI/R rat models (Supplementary Figure 1B). Furthermore, to investigate whether USP22 is involved in MI/R myocardial injury, SD rats were subjected to 30 min of ischemia and 3 or 24 h of reperfusion. RT-qPCR and Western blot analysis were further adopted to detect the expression patterns of USP22 in myocardial tissue following MI/R injury. The results revealed that the expression of USP22 decreased after 3 h of reperfusion, and decreased further after 24 h of reperfusion (Figure 1A). Immunohistochemistry was additionally performed to detect the expression patterns of USP22 in the myocardial tissue of rats, and as expected, the expression of USP22 in the myocardial tissue of the MI/R rats was found to be reduced (Figure 1B). Accordingly, we hypothesized that USP22 could be involved in the development of MI/R injury.

RETRACTED

**FIGURE 1:** USP22 attenuates MI/R injury in rats (*n* = 12/group). **(A)** RT-qPCR and Western blot analysis detection of USP22 expression in the myocardial tissue of the sham-operated and MI/R rats 3 and 24 h after MI/R. **(B)** Immunohistochemical detection of USP22 expression in myocardial tissue 24 h after MI/R. **(C)** RT-qPCR and Western blot analysis detection of the expression of USP22 in myocardial tissue 24 h after MI/R in rats. **(D)** TCC staining detection and ImageJ quantification of the area of myocardial infarction following USP22 overexpression. **(E)** Detection of rat serum CPK and LDH levels following USP22 overexpression. * indicates comparison with the sham-operated rats, *p* < 0.05; # indicates comparison with the MI/R rats treated with oe-NC, *p* < 0.05. One-way ANOVA followed by Tukey posttest was used for comparison between multiple sets of data. NC, negative control; MI/R, myocardial ischemia–reperfusion; CPK, creatine phosphokinase; LDH, lactate dehydrogenase.

Subsequently, USP22 was overexpressed in rat myocardial tissues by intravenous injection of adenovirus and undergone I/R or sham-operated surgery. The results of RT-qPCR and Western blot analysis verified the overexpression efficiency of USP22 in myocardial tissue (Figure 1C). In addition, TTC staining results demonstrated that the hearts in the sham-operated rats were normal, whereas USP22 overexpression led to smaller area of myocardial infarction in the MI/R rats (Figure 1D). As expected, CPK and LDH levels were markedly reduced in the USP22-overexpressed MI/R rats compared with MI/R rats at 24 h after injury (Figure 1E). Collected, these findings indicated that overexpression of USP22 attenuated the MI/R injury in rats.

### USP22 Overexpression Inhibits Myocardial Death Caused by Ferroptosis

In the subsequent experiments, overexpression or knock down experiments were performed in H9C2 cardiomyocytes, and confirmed the transfection efficiency of USP22 by RT-qPCR and Western blot analysis (Supplementary Figure 2A). Next, IR models were established in cardiomyocytes, and assessed the content of LDH in the supernatant. It was found that the LDH was reduced in cells after USP22 overexpression, indicating reduced myocardial cell death, whereas opposite trends were noted in the cells after USP22 knockdown (Figure 2A). Subsequently, MTT assay was adopted to detect myocardial cell viability, which revealed that cell viability was increased in the cells with USP22 overexpression compared with the oe-NC-treated cells, whereas cell viability was decreased in the cells with USP22 knockdown compared with the sh-NC-treated cells (Figure 2B). Based on the above findings, we speculated that USP22 could influence the process of cell death. Therefore, Z-VAD-FMK (cell necrosis inhibitor), Nercrostain-1 (apoptosis inhibitor), and Liproxstatin-1 (ferroptosis inhibitor) were adopted to treat USP22 knockdown cells and then measured LDH content, which demonstrated that only Liproxstatin-1 inhibited cell death induced by USP22 knockdown (Figure 2C). Additionally, GSH, Reactive oxygen species, lipid peroxidation, and iron accumulation are regarded as important indicators of activated ferroptosis signaling pathway. Therefore, the aforementioned factors were measured after knocking down or overexpressing USP22 in cells, which demonstrated that USP22 overexpression increased GSH, while decreasing reactive oxygen species production, lipid peroxidation, and iron accumulation, whereas opposite trends were noted after USP22 knockdown in cells (Figure 2D). Furthermore, flow cytometry was conducted to determine cell apoptosis, displaying no significant difference in cell apoptosis in response to the oe-USP22 + sh-NC or oe-NC + sh-USP22 compared with oe-NC + sh-NC (Supplementary Figure 2B). The above results indicated that USP22 elevation inhibited ferroptosis-induced myocardial cell death.

RETRACTED

**FIGURE 2:** USP22 elevation inhibits ferroptosis-induced myocardial cell death. **(A)** LDH level detected in the supernatant of H9C2 cells. **(B)** MTT detection of H9C2 cell viability. **(C)** Detection of LDH levels in the supernatant of H9C2 cells after treatment with different inhibitors. **(D)** Detection of GSH, reactive oxygen species, lipid peroxidation, and accumulation of iron. * indicates comparisons with the cells treated with oe-NC; # indicates comparisons with cells with sh-NC, *p* < 0.05. One-way ANOVA followed by Tukey posttest was used for comparison between multiple sets of data. NC, negative control; GSH, glutathione.

### USP22 Inhibits SIRT1 to Regulate Ferroptosis-Induced Cardiomyocyte Death

A previous study has shown that USP22 possesses the ability to stabilize SIRT1 by the process of deubiquitination (Lin et al., 2012). To better understand its underlying mechanism, the expression patterns of SIRT1 in myocardial tissues after MI/R injury were detected by RT-qPCR and Western blot analysis, which demonstrated that SIRT1 expression decreased after 3 h of reperfusion, and decreased further after 24 h of reperfusion (Figure 3A). To test whether the expression of SIRT1 could be affected by USP22, USP22 expression in H9C2 cells was overexpressed or knocked down, and Western blot analysis revealed that SIRT1 expression increased after USP22 overexpression, while exhibiting a decrease after USP22 knockdown (Supplementary Figure 3A). Meanwhile, the interaction between USP22 and SIRT1 was validated using a ChIP assay (Figure 3B). Furthermore, the changes in ubiquitination levels of SIRT1 after USP22 overexpression were examined through ChIP assay, which revealed that USP22 overexpression decreased the ubiquitination level of SIRT1 (Figure 3C).

RETRACTED

**FIGURE 3:** Deubiquitination of USP22 stabilizes SIRT1 expression to further inhibit ferroptosis-induced cell death. **(A)** RT-qPCR and Western blot analysis detection of SIRT1 expression in myocardial tissues in rats after 3 and 24 h of MI/R (*n* = 12/group). **(B)** ChIP assay of the binding between USP22 and SIRT1. **(C)** ChIP assay of USP22’s ubiquitination effect on SIRT1. **(D)** Detection of GSH, reactive oxygen species, lipid peroxidation, and iron accumulation following overexpression or knockdown of SIRT1. **(E)** Detection of GSH, reactive oxygen species, lipid peroxidation, and iron accumulation following USP22 overexpression and SIRT1 knockdown. * indicates *p* < 0.05 compared with sham-operated rats, MI/R rats injected with oe-NC or oe-NC + sh-NC; # indicates *p* < 0.05 compared with rats received 3-h reperfusion, MI/R rats injected with sh-NC or oe-USP22 + sh-NC. One-way ANOVA followed by Tukey posttest was used for comparison between multiple sets of data. NC, negative control; GSH, glutathione.

Additionally, to better understand the role of USP22-SIRT1 axis in ferroptosis-induced cell death, the effects of overexpression or knockdown of SIRT1 on ferroptosis signaling pathway were examined using Western blot analysis (Supplementary Figure 3B). The results displayed that overexpression of SIRT1 led to increased GSH in the downstream of ferroptosis, in addition to a reduction in reactive oxygen species production, lipid peroxidation, and iron accumulation, whereas opposite trends were observed in response to SIRT1 silencing (Figure 3D). Further, cells were treated with oe-USP22 + sh-SIRT1 (Supplementary Figure 3A), and results demonstrated that SIRT1 knockdown reversed the effect of USP22 overexpression on increased GSH, reduced reactive oxygen species, lipid peroxidation, and iron accumulation (Figure 3E), highlighting that SIRT1 served as a mediator of USP22 to regulate ferroptosis-induced cardiomyocyte cell death.

### SIRT1 Inhibits Ferroptosis-Induced Myocardial Cell Death Through p53/SLC7A11 Axis

Prior studies have noted that p53 contributes to aging and cardiovascular stress-induced cell death, and SIRT1 can potentially regulate the acetylation of p53 and its downstream signaling cascade (Zhang et al., 2014). Thus, the expression patterns of p53 in myocardial tissues after MI/R injury were detected with RT-qPCR and Western blot analysis, which revealed that the expression of p53 increased after 3 h of reperfusion, and increased further after 24 h of reperfusion (Figure 4A). Moreover, SIRT1 was overexpressed or knocked down in H9C2 cells (Supplementary Figure 4A), and then p53 acetylation levels were detected by Western blot analysis, which demonstrated that SIRT1 overexpression reduced p53 acetylation and protein levels, whereas opposite trends were observed upon SIRT1 knockdown (Figure 4B). As expected, p53 depletion increased GSH, but decreased reactive oxygen production, lipid peroxidation, and iron accumulation, whereas contradictory trends were noted upon p53 overexpression (Figure 4C), suggesting that p53 promoted ferroptosis-induced cell death.

RETRACTED

**FIGURE 4:** SIRT1 inhibits ferroptosis-induced myocardial cell death by regulating p53/SLC7A11 expression. **(A)** RT-qPCR and Western blot analysis detection of p53 expression in myocardial tissue after 3 and 24 h of MI/R (*n* = 12/group). **(B)** Effect of SIRT1 on acetylation level of p53 detected by ChIP assay. **(C)** Detection of GSH, reactive oxygen species, lipid peroxidation, and iron accumulation upon p53 overexpression or knockdown. **(D)** RT-qPCR and Western blot analysis detection of SLC7A11 expression in myocardium tissue of the sham-operated rats after 3 and 24 h MI/R (*n* = 12/group). **(E)** ChIP assay of the binding relationship between p53 and SLC7A11. **(F)** Western blot analysis detection of SIRT1, p53, and SLC7A11 protein expression in H9C2 cells following overexpressing SIRT1 and knocking down SLC7A11. **(G)** Detection of GSH, reactive oxygen species, lipid peroxidation, and iron accumulation following overexpressing SIRT1 and knocking down SLC7A11. * indicates *p* < 0.05 compared with sham-operated rats, rats received 3 h reperfusion or MI/R rats injected with oe-NC; # indicates *p* < 0.05 compared with rats received 3 h reperfusion or MI/R rats injected with sh-NC or oe-SIRT1 + sh-NC. One-way ANOVA followed by Tukey posttest was used for comparison between multiple sets of data. NC, negative control; MI/R, myocardial ischemia–reperfusion; GSH, glutathione.

Moreover, p53 has been reported to regulate the expression of SLC7A11, a key protein in the ferroptosis signaling pathway (Wang et al., 2020). Therefore, the expression patterns of SLC7A11 in myocardial tissues after MI/R injury were detected by RT-qPCR and Western blot analysis. The expression of SLC7A11 was found to be decreased after 3 h of reperfusion, and further decreased after 24 h of reperfusion (Figure 4D). In addition, Western blot analysis results demonstrated that p53 overexpression inhibited the expression of SLC7A11, whereas p53 suppression brought about the opposite results, indicating that p53 could negatively target SLC7A11 (Supplementary Figure 4B), which was further confirmed by ChIP assay, displaying that p53 can bind to the promoter of SLC7A11 (Figure 4E). Consistently, Western blot analysis results revealed that the expression of SLC7A11 increased when SIRT1 was overexpressed, while being unchanged in response to oe-SIRT1 + oe-p53 (Figure 4F). In the subsequent experiments, myocardial cells were treated with oe-SIRT1 + oe-NC, or oe-SIRT1 + sh-SLC7A11 (Figure 4G), and found that overexpression of SIRT1 resulted in increased consumption of GSH, in addition to reduced reactive oxygen species production, lipid peroxidation, and iron accumulation, whereas these trends were reversed by SLC7A11 knockdown (Figure 4G). Moreover, flow cytometry assessment of cell apoptosis exhibited that cell apoptosis exhibited no significant differences following the treatments of oe-NC + sh-NC, oe-USP22 + sh-SIRT1, oe-SIRT1 + sh-NC, and oe-SIRT1 + sh-SLC7A11 (Supplementary Figure 5). Coherently, SIRT1 inhibited ferroptosis-induced myocardial cell death through p53/SLC7A11.

RETRACTED

### USP22 Protects Against MI/R Injury Through SIRT1/p53/SLC7A11 Axis *in vivo*

Based on the above-mentioned results, it was speculated that USP22 protects against MI/R injury through the SIRT1/p53/SLC7A11 axis. Therefore, MI/R rats were injected with adenovirus vectors containing oe-USP22 + sh-NC, oe-USP22 + sh-SIRT1, oe-USP22 + sh-SLC7A11, and oe-NC + sh-NC. Afterward, the expression patterns of USP22, SIRT1, p53, and SLC7A11 in the myocardial tissue of rats were detected by Western blot analysis, which revealed that when USP22 was overexpressed, SIRT1 and SLC7A11 expressions were increased, and that of p53 was reduced. Treatment with oe-USP22 + sh-SIRT1 brought about increased USP22 and p53 expressions, but decreased SIRT1 and SLC7A11 expression, whereas opposite trends were noted upon oe-USP22 + sh-SLC7A11 treatment (Figure 5A). Moreover, the extent of MI was determined by Evans blue and TTC staining, which illustrated similar ratios of area at risk (AAR) to left ventricular area in the MI/R rats treated with oe-USP22, oe-USP22 + sh-SLC7A11, and oe-USP22 + SIRT1. However, compared with MI/R rats treated with oe-USP22 + sh-SLC7A11 or oe-USP22 + SIRT1, the ratio of infarct area to AAR in rats treated with oe-USP22 was found to be reduced by approximately 63% (Figure 5B). As expected, CPK and LDH levels in oe-USP22-treated rats were significantly lower than those in the rats following treatment of oe-USP22 + sh-SLC7A11 or oe-USP22 + SIRT1 after 24 h of MI/R (Figure 5C). In addition, hematoxylin–eosin (H&E) staining results demonstrated that the myocardial tissues of the sham-operated rats were regularly arranged without necrosis. Compared with sham-operated rats, the MI/R rats were observed to exhibit myocardial fiber deformation and disturbance accompanied by inflammatory cell infiltration, and myocardial cell swelling, whereas these conditions were alleviated in response to oe-USP22, whereas the conditions in the rats following treatment of oe-USP22 + sh-SLC7A11 or oe-USP22 + SIRT1 remained unchanged (Figure 5D). Moreover, hemodynamic measurements were conducted on rats, which revealed that compared to MI/R rats with USP22 overexpression alone, the rats with treatment of oe-USP22 + sh-SLC7A11 or oe-USP22 + SIRT1 exhibited a reduction in maximum pressure, ejection fraction, and maximum pressure rate (dP/dT max) (Figure 5E), highlighting the exacerbated cardiac function of rats. Taken together, these findings indicated that USP22 protected against MI/R injury through the SIRT1/p53/SLC7A11 axis *in vivo*.

RETRACTED

**FIGURE 5:** USP22 protected against MI/R injury through SIRT1/p53/SLC7A11 axis in rats. We injected MI/R rats with adenovirus vectors containing MI/R + oe-USP22 + sh-NC, MI/R + oe-USP22 + sh-SIRT1, MI/R + oe-USP22 + sh-SLC7A11, or MI/R + oe-NC + sh-NC (*n* = 6/group). **(A)** USP22, SIRT1, p53, and SLC7A11 expression in myocardial tissue of rats detected by Western blot analysis. **(B)** TCC staining detection and ImageJ quantification of the area of myocardial infarction. **(C)** Serum CPK and LDH levels of rats detection in rats. **(D)** H&E staining of myocardial tissue pathological changes of rats. **(E)** Detection of cardiac functions of rats, including maximum pressure, ejection fraction, and maximum pressure increasing rate. * represents comparisons with the sham-operated rats, *p* < 0.05; # represents comparisons with the MI/R rats injected with oe-NC + sh-NC, *p* < 0.05; & represents comparisons with the MI/R rats injected with oe-USP22 + sh-NC, *p* < 0.05. One-way ANOVA followed by Tukey posttest was used for comparison between multiple sets of data. NC, negative control; MI/R, myocardial ischemia–reperfusion; CPK, creatine phosphokinase; LDH, lactate dehydrogenase.

## Discussion

The past few decades have witnessed the integration of various measures to minimize MI/R injury in clinical settings (Ibanez et al., 2015). Moreover, years of continuous investigations have summarized myocardial reperfusion injury in the following four defined categories: reperfusion-induced arrhythmias, myocardial stunning, microvascular obstruction, and lethal myocardial reperfusion injury, among which the first two injuries proved to be reversible while the latter two being irreversible in nature (Hausenloy and Yellon, 2013). In particular, reperfusion-caused death of cardiomyocytes, a feature of ischemic period, is characterized as the last form of injury, leading us to figure out the potential role of cell death mechanism underlying MI/R injury processes. Our findings demonstrated that USP22 overexpression inhibited ferroptosis-induced cardiomyocyte death to protect against MI/R injury *via* the SIRT1/p53/SLC7A11 pathway using *in vivo* and *in vitro* experimentation.

RETRACTED

Initially, findings in the current study revealed that USP22 was poorly expressed in myocardial tissues after the occurrence of MI/R injury, whereas USP22 elevation attenuated MI/R injury by enhancing cardiomyocyte viability and lessening ferroptosis-induced cell death as evidenced by increased GSH, decreased reactive oxygen species, lipid peroxidation, and iron accumulation. Consistently, the up-regulation of USP22 has been proven to promote intestinal cell proliferation and tissue regeneration following I/R or hypoxia/reoxygenation, thus exerting a similar protective function on intestinal I/R injury (Ji et al., 2019). Ferroptosis is involved in the oxygen-glucose deprivation/reoxygenation-induced Sertoli cell death, commonly characterized by elevated iron and lipid reactive oxygen species levels in I/R injury and depleted GSH (Li et al., 2018).

Moreover, we found that USP22 inhibited the SIRT1 gene to regulate ferroptosis-induced cardiomyocyte death. This is supported by the findings of Lin et al. (2012) which stated that USP22 functions as a specific deubiquitinase of SIRT1. Deubiquitinating enzymes (DUBs) possess the ability to invert ubiquitination of aimed proteins, maintaining an equalized balance between deubiquitination and ubiquitination of targeted proteins to preserve cell homeostasis (Tanguturi et al., 2020). Deubiquitinases belong to proteases, which could play important roles in modulating the stability, activity, and translocation of targeted protein by removing its ubiquitins (Xiao et al., 2016). For instance, Ubiquitin Specific Protease 49 (USP49) was previously shown to interact with apolipoprotein B mRNA editing enzyme catalytic polypeptide-like 3G (APOBEC3G, A3G) to rapidly remove its ubiquitin, which efficiently stabilizes A3G and augments A3G protein expression levels, and further inhibited the replication of HIV-1 (Pan et al., 2019). Meanwhile, SIRT1 has been reported to exert a protective role in myocardia injury (Fu et al., 2017), whereas our findings demonstrated that SIRT1 expression was repressed in myocardial tissue after MI/R injury, whereby its elevation reduced the extent of MI/R injury by enhancing cardiomyocyte viability and diminishing ferroptosis-induced cell death. Furthermore, another study revealed that treatment with resveratrol, a SIRT1 activator, weakened cardiac function and reduced cardiomyocyte apoptosis in the context of diabetic cardiomyopathy, which supports our findings in regard to SIRT1 elevation (Guo et al., 2015). In addition, our findings consistently confirmed that USP22 can stabilize the expression of SIRT1 by deubiquitination to inhibit ferroptosis-induced cell death in cardiomyocytes.

RETRACTED

During subsequent experimentation, we further uncovered that SIRT1 inhibited ferroptosis-induced myocardial cell death through the p53/SLC7A11 axis. This is noteworthy as one previous study revealed that TQ confers protection against MI/R injury through activation of the SIRT1 signaling pathway to reduce mitochondrial oxidative stress damage and cardiomyocyte apoptosis by inhibiting p53 acetylation (Lu et al., 2018). Furthermore, another study also proposed that p53 (especially acetylation-defective mutant p53) positively regulates ferroptosis by inhibiting the SLC7A11 expression to promote the production of reactive oxygen species (Xie et al., 2016). SLC7A11 encodes an element of the cystine/glutamate antiporter complex, which is connected by disulfide-linked heterodimerization of both SLC-3A2 and -7A11 (Jiang et al., 2015a). Recently, further investigations have also revealed that reactive oxygen species–induced ferroptosis could potentially be suppressed by high levels of SLC7A11 (Jiang et al., 2015b). As a result, these implications hinted at us that p53/SLC7A11 could be a potential axis governing the ferroptosis activity on cardiomyocytes of downstream of SIRT1.

To summarize, the current study revealed that USP22 deubiquitination could stabilize the expression levels of SIRT1. Moreover, SIRT1 overexpression could bring about a reduction in p53 acetylation and protein levels, whereas p53 suppression could elevate the SLC7A11 levels. Collectively, this mechanism inhibits ferroptosis-induced cardiomyocyte death in MI/R injury (Figure 6). Our findings could provide a novel therapeutic target for MI/R injury treatment. Our study incorporated the use of both *in vivo* model and *in vitro* models, and accompanied by a wide range of methodology. However, further studies should be performed in a clinical setting. Besides, in this investigation, we focused on only one selected main pathway (the SIRT1/p53/SLC7A11 axis), and the effect of USP22 on other pathways should also be explored in the future.

**FIGURE 6:** Mechanism. USP22 deubiquitination stabilizes, and upregulates the expression level of SIRT1. SIRT1 overexpression leads to a reduction of p53 acetylation and protein level to elevate SLC7A11 level. Collectively, this mechanism inhibits ferroptosis-induced cardiomyocyte death so as to protect against MI/R injury.

RETRACTED

## Data Availability Statement

All datasets presented in this study are included in the article/Supplementary Material.

## Ethics Statement

The animal study was reviewed and approved by the Animal Experiment Ethics Committee from the Second Hospital of Hebei Medical University.

## Author Contributions

SM and LS wrote the manuscript. WW and JW conceived and designed the experiments. ZS analyzed the data. JR collected and provided the sample for this study. All authors have read and approved the final submitted manuscript.

## Conflict of Interest

The authors declare that the research was conducted in the absence of any commercial or financial relationships that could be construed as a potential conflict of interest.

## Supplementary Material

FIGURE S1 MI/R injury models in rats were successfully established. **(A)** TCC staining detection and Image J quantification of the area of myocardial infarction. **(B)** Serum CPK and LDH levels in rats; NC, negative control; CPK, creatine phosphokinase; LDH, lactate dehydrogenase.

FIGURE S2 Verification of transfection efficiency in H9C2 cells and its effect on cell apoptosis. **(A)** RT-qPCR and Western blot analysis validation of transfection efficiency in H9C2 cells. **(B)** Cell apoptosis determined using flow cytometry. ^∗^Represents comparisons with the cells treated with oe-NC, *p* < 0.05; # represents comparisons with the cells treated with sh-NC, *p* < 0.05; One-way ANOVA followed by Tukey’s posttest was used for comparison between multiple sets of data. NC, negative control.

FIGURE S3 Verification of transfection efficiency in H9C2 cells of USP22/SIRT1 in cardiomyocytes. **(A)** Western blot analysis detection of SIRT1 expression in H9C2 cells with USP22 overexpressed or knocking down. **(B)** Western blot analysis detection of SIRT1 expression in H9C2 cells with SIRT1 overexpressed or knocking down. ^∗^Represents comparisons with the cells treated with oe-NC or oe-NC + sh-NC, *p* < 0.05; # represents comparisons with the cells treated with sh-NC, *p* < 0.05; One-way ANOVA followed by Tukey’s posttest was used for comparison between multiple sets of data. NC, negative control.

FIGURE S4 Verification of transfection efficiency of p53 in H9C2 cells and its effects on SLC7A11. **(A)** Western blot analysis validation of p53 transfection efficiency in H9C2 cells; **(B)** Western blot analysis detection of SLC7A11 expression in H9C2 cells with p53 overexpressed or knocking down. ^∗^Represents comparisons with the cells treated with oe-NC, *p* < 0.05; # represents comparisons with the cells treated with sh-NC, *p* < 0.05; One-way ANOVA followed by Tukey’s posttest was used for comparison between multiple sets of data. NC, negative control.

RETRACTED

FIGURE S5 The effects of SIRT1/SLC7A11 on H9C2 cells. Cell apoptosis determined using flow cytometry. One-way ANOVA followed by Tukey’s posttest was used for comparison between multiple sets of data. NC, negative control.

FIGURE S6 Experimental scheme.
